This article has been retracted.

# Incidence of Adverse Effects of Propofol for Procedural Sedation/Anesthesia in the Pediatric Emergency Population: A Systematic Review and Meta-Analysis

**DOI:** 10.1155/2021/3160154

**Published:** 2021-12-23

**Authors:** Pengfei Guo, YingChun Ran, Xiaoxiao Ao, Qing Zou, Liping Tan

**Affiliations:** Department of Emergency, Children's Hospital of Chongqing Medical University, Chongqing 400014, China

## Abstract

**Background:**

To investigate the incidence of adverse effects of propofol among pediatric population for sedation or anesthesia.

**Methods:**

We performed Cochrane Library, PubMed, CNKI, VIP, and Wanfang databases to research relevant literature. We did sensitivity analysis to assess the incidence of adverse effects of propofol among pediatric population for sedation or anesthesia.

**Results:**

In 132 studies, eight RCTs were included in this analysis. The result showed that adverse events (bradypnea, hypotension, hypertension, and apnea) were significantly improved in the pediatric emergency population in the propofol group, but it had no effect on the incidence of cough attacks, desaturation, agitation, stridor, and laryngospasm. Furthermore, the subgroup analysis showed that those who received propofol for had decreased adverse effects compared with the patients who received ketamine treatment (SMD = 0.44, 95%CI = [0.28, 0.67], *I*^2^ = 0%, and *P* = 0.0002), which demonstrated that propofol could decrease the incidence of adverse effects compared with ketamine and ketofol.

**Conclusions:**

The study demonstrated that propofol may decrease the incidence of bradypnea, hypotension, hypertension, and apnea, but it had no effect on the incidence of cough attacks, desaturation, agitation, stridor, and laryngospasm. Furthermore, more large RCTs are needed to assess incidence of adverse effects of propofol among pediatric population.

## 1. Introduction

Pediatric emergency treatment is often accompanied by trauma or pain. Some painful or uncomfortable procedures may be necessary during emergency treatment, and emergency physicians are needed to provide safe and effective analgesia and sedation for children [1, 2]. Moreover, local anesthesia and regional anesthesia together with appropriate safety procedures should be used for sedation to avoid aggravation of pain to ensure that the pediatric population will not suffer long-term or extra pain in emergency [3]. At present, the commonly used procedural sedative and analgesic drugs in pediatric emergency include chloral hydrate, nitrous oxide, benzodiazepines, dexmedetomidine, propofol, ketamine, morphine, ibuprofen, fentanyl, ketoalcohol, and methoxyfluorane [4–10]. Nevertheless, the poor effect of pediatric procedural sedation/anesthesia in the emergency department is due to the side effects and adverse reactions of drugs are not clear to clinicians [11, 12].Propofol is a sedative-hypnotic agent widely used for procedural sedation [13]. It is a kind of powerful hypnotic and sedative drug. It exerts hypnotic effect by activating the central inhibitory neurotransmitter GABA, and it has the characteristics of rapid onset and recovery [14]. The advantages of propofol include rapid onset, quick and predictable recovery time, and antiemetic effects. Disadvantages include dose-dependent hypotension, bradycardia, respiratory depression, and pain with injection [15–18]. In addition, propofol does not provide analgesia [19]. However, whether propofol is used for sedation in children is still controversial. Schacherer et al. [20] compared the safety and effectiveness of propofol and dexmedetomidine for mild sedation in children. The results showed that the average recovery time of propofol (34.3 min) was significantly lower than dexmedetomidine (65.6 min). 9.7% of children needed respiratory support, including balloon ventilation of 2.3%, respiratory obstruction of 1.1%, and decrease of oxygen saturation of 1.6%, and no children needed tracheal intubation.

To determine incidence of adverse effects of propofol among pediatric population, we did systematic review and meta-analysis.

## 2. Materials and Methods

### 2.1. Search Strategy

This study based on Cochrane Handbook [21], and it published conforming to the meta-analysis statement [22]. We researched the databases: Cochrane Library, PubMed, CNKI, VIP, and Wanfang. The search strategy was as follows: ((“Propofol”) AND(“Procedural Sedation” OR “Anesthesia”) AND (“Pediatric” And “Emergency department”)).

### 2.2. Inclusion and Exclusion Criteria

The inclusion criteria are as follows: (a) studies that assessed adverse effects of propofol, (b) studies that reported baseline and follow-up data of adverse events or sufficient information which allowed for the calculation of adverse events, and (c) RCTs.

The exclusion criteria are as follows: (a) observational study, (b) animal research, (c) research of other new drug intervention, (d) the outcome indicators of literature application cannot be extracted or calculated, and (e) the data were repeatedly published.

### 2.3. Data Extraction and Quality Assessment

Two researchers screened the study, respectively, and checked the selected researches in accordance with the inclusion and exclusion criteria. When there was any objection to a certain research, the third researcher was consulted to finally determine the selected researches. The flow chart of literature screening is shown in Figure 1. Two researchers blindly collected the capital data (first author, year of publication, research method, research object, sample size, average age, and course of treatment) and outcome indicators (echocardiographic indicators, mortality, rehospitalization rate due to heart failure, symptomatic hypotension, renal function injury rate, hyperkalemia, and incidence of vascular edema). The bias risk assessment tool in Cochrane Handbook for systematic review of interventions (version 5.1.0) was used to evaluate the quality of the included studies. The results of the quality assessment are shown in Figure 2.

### 2.4. Statistical Analysis

The Review Manager Software (RevMan, version 5.2 from the Cochrane Collaboration) was used for data analysis and statistics of all outcome indicators. According to the heterogeneity test results, the effect model was determined. *I*^2^ ≥ 50% indicates greater heterogeneity, and the RE model was selected; *I*^2^ ≤ 50% indicates that the heterogeneity is within the acceptable range, and the fixed effect model (FE) is selected. When *P* < 0.05, it was considered that there were significant differences in the changes of each outcome index. Subgroup analysis was used to identify the source of heterogeneity, and sensitivity analysis was used to assess the impact of individual studies on the overall results.

## 3. Results

### 3.1. Flow Chart of Study Selection

A diagram of the study selection is shown in Figure 1. As the result, eight RCTs [23–30] were included in this studies: three RCTs comparing propofol with sevoflurane [24, 28, 30], three comparing propofol with ketamine [25, 26, 29], one comparing propofol with ketofol for procedural sedation/anesthesia in the pediatric emergency population [27], and one comparing propofol with remifentanil [23]. Furthermore, among the eight studies eligible for the meta-analysis, a total of 945 subjects were enrolled. Among them, 481 subjects were randomized to receive propofol.

### 3.2. Characteristics of Included Studies

The characteristics are seen in Tables 1 and 2. 945 population were enrolled. 481 patients received propofol. Three studies were performed in western countries. Three RCT studies compared propofol with sevoflurane for procedural sedation/anesthesia in the pediatric emergency population [24, 28, 30], three compared propofol with ketamine [25, 26, 29], one compared propofol with ketofol [27], and one compared propofol with remifentanil [23]. Figure 2 shows the risk of bias of eight studies [23–30]. The included studies were assessed moderate to high of bias.

### 3.3. Pooled Analysis

The study demonstrated that adverse events (bradypnea, hypotension, hypertension, and apnea) were significantly improved in the pediatric emergency population in the propofol group (random effect model, Figure 3). The incidence of bradypnea hypotension, hypertension, and apnea was decreased compared to the control group (*P* < 0.05). This pooled analysis did not show (*I*^2^ = 0% and *P* = 0.53).

### 3.4. Subgroup Analysis

We conducted the subgroup analysis compared the differences between ketamine, ketofol, and sevoflurane (Figure 4). In this subgroup analysis, the results demonstrated that those who received propofol for had decreased adverse effects compared with the patients who received ketamine treatment (SMD = 0.44, 95%CI = [0.28, 0.67], *I*^2^ = 0%, and *P* = 0.0002). And the overall effect (SMD = 0.44, 95%CI = [0.28, 0.67], *I*^2^ = 0%, and *P* = 0.0002) demonstrated that propofol could decrease the incidence of adverse effects compared with ketamine and ketofol.

### 3.5. Sensitivity Analysis and Publication Bias

Sensitivity analysis revealed that removal of any one study from the analysis did not subvert the results of the pooled analysis (data not shown). Similarly, excluding two studies enrolling cough attack event [23, 25] did not influence our primary analyses for adverse effects (SMD, 0.24; 95% CI: 0.03-0.45; and *P* = 0.02). Therefore, the outcome of the pooled analysis can be regarded with a higher degree of certainty. Furthermore, we constructed funnel plots to evaluate publication bias. The funnel plots (Figure 5) showed no publication bias.

## 4. Discussion

The study showed that adverse events (bradypnea, hypotension, hypertension, and apnea) were significantly improved in the pediatric emergency population in the propofol group; furthermore, the study did not show heterogeneity (*I*^2^ = 0% and *P* = 0.53).

A total of eight of RCTs were high-quality article. The combined results showed that compared with other sedative drugs, propofol had decreased the incidence of bradypnea, hypotension, hypertension, and apnea, but it had no effect on the incidence of cough attacks, desaturation, agitation, stridor, and laryngospasm. At present, there are few large-scale clinical trials of propofol, and there is a lack of clinical data. Moreover, more studies are needed to assess the safety of propofol among pediatric.

Our study showed that propofol has decreased the incidence of bradypnea, hypotension, hypertension, and apnea. The result revealed that patients who with treatment of propofol decreased the incidence of other respiratory and circulatory diseases. This may explained that propofol had effect on airway smooth muscle reflexes [31]. Previous researches in the pediatric did not demonstrate the relationship between side effects and propofol/ketamine [32–37]. Pain with intravenous administration is an adverse effect of propofol [38–41].

The study has some weakness. Firstly, it is the number of studies included. We included eight studies, and most of the studies were single-center studies. In addition, we did not analyze the more adverse events in subgroup. Therefore, we could not comprehensively summarize the adverse events. Moreover, other measurements such as individual differences of the pediatric serve as confounding factors. Finally, this review cannot rule out statistical differences because of the included single-center studies. Therefore, more RCTs should be conducted to assess the incidence of adverse events of propofol.

## 5. Conclusion

In conclusion, this review showed the incidence of adverse events of propofol for procedural sedation/anesthesia. It demonstrated that it decreased incidence of adverse events of propofol for the pediatric emergency population. Furthermore, there was no effect on the incidence of cough attacks, desaturation, agitation, stridor, and laryngospasm. The data suggest that propofol may decrease the incidence of bradypnea, hypotension, hypertension, and apnea among the pediatric emergency population. More clinical trials are needed to assess the incidence of adverse effects of propofol among pediatric population for procedural sedation/anesthesia in the emergency department.

## Figures and Tables

**Figure 1:** Flow diagram of the literature search.

**Figure 2:** The risk of bias of randomized trials included in the meta-analysis.

**Figure 3:** Forest plot for the meta-analysis of adverse effects.

**Figure 4:** Subgroup analysis compared the differences between propofol with ketamine, ketofol, and sevoflurane.

**Figure 5:** The funnel plots for cough attacks.

**Table 1:** Characteristics of the 8 studies in the meta-analysis.

Author Year	Country	Age (EG vs. CG) Mean ± SD	Size EG/CG	Types of studies and intervention	Doses
Chen 2013 [23]	China	2 ± 8.7 vs. 2.2 ± 6.0	25/25	RCT comparing the use of propofol remifentanil	Propofol 8.3 *μ*g/ml
Weng 2020 [24]	China	8.9 ± 2.9 vs. 9.3 ± 3.8	60/60	RCT comparing the use of propofol+sevoflurane	Propofol 9-15 mg/(kg/h)
Erden 2009 [25]	Turkey	8.93 ± 4.0 vs. 6.97 ± 3.8	30/30	RCT comparing the use of propofol+ketamine	Propofol 0.5 mg/kg
Weisz 2017 [26]	American	8.3 ± 6.3 vs. 9.3 ± 5.5	96/87	RCT comparing the use of propofol+ketamine	Propofol 1.0 mg/kg
Mittal 2013 [27]	India	4.6 ± 1.32 vs. 4.4 ± 1.62	20/20	RCT comparing the use of propofol+Ketofol	Propofol 1.0 mg/kg
Wu 2020 [28]	China	5.3 ± 2.3 vs. 6.1 ± 3.1	37/36	RCT comparing the use of propofol+sevoflurane	Propofol 1.0 mg/kg
Schmitz 2018 [29]	Switzerland	3.67 ± 1.6 vs. 3.91 ± 2.1	167/164	RCT comparing the use of propofol+ketamine	Propofol 1.0 mg/kg
Hasani 2013 [30]	Serbia	4.0 ± 1.5 vs. 4.0 ± 1.6	46/42	RCT comparing the use of propofol+sevoflurane	Propofol 9-13 mg/(kg/h)

**Table 2:** Characteristics of the 8 included studies on adverse events.

Author	Country	Age	Adverse events	Blinding
Chen 2013 [23]	Eastern	<18	Cough attacks, oral aspiration, desaturation, bradypnea, hypotension, hypertension, bradycardia	Double-blind
Weng 2020 [24]	Eastern	<18	Cough attacks, hypotension, hypertension, bradycardia, stridor	Double-blind
Erden 2009 [25]	Western	<18	Agitation, tachycardia, nystagmus, bradypnea, hypotension, hypertension	Double-blind
Weisz 2017 [26]	Western	<18	Oxygen desaturation, apnea, cardiovascular events, nausea, vomiting/retching, unpleasant recovery reaction	Double-blind
Mittal 2013 [27]	Eastern	<18	Apnea, desaturation, stridor, coughing, laryngospasm	Double-blind
Wu 2020 [28]	Eastern	<18	Hypoxia, agitation	Double-blind
Schmitz 2018 [29]	Western	<18	Agitation, stridor, laryngospasm, apnea	Double-blind
Hasani 2013 [30]	Eastern	<18	Hypotension, bradycardia, laryngospasm, hypertension, postoperative nausea, postoperative vomiting, cough attacks	Double-blind

## Data Availability

The data used in the article can be obtained from Cochrane Library, PubMed, CNKI, VIP, and Wanfang databases.
